# The adipokine vaspin reduces apoptosis in human hepatocellular carcinoma (Hep-3B) cells, associated with lower levels of NO and superoxide anion

**DOI:** 10.1186/s40360-019-0334-6

**Published:** 2019-09-11

**Authors:** Magdalena Skonieczna, Dorota Hudy, Tomasz Hejmo, Rafal J. Buldak, Małgorzata Adamiec, Michal Kukla

**Affiliations:** 1 Systems Engineering Group, Silesian University of Technology, Institute of Automatic Control, 16 Akademicka Street, 44-100 Gliwice, Poland; 2 Biotechnology Centre, Silesian University of Technology, Krzywoustego 8, 44-100 Gliwice, Poland; 3 Department of Biochemistry, Medical University of Silesia, School of Medicine with the Division of Dentistry, Jordana 19, 41-808 Zabrze, Poland; 4 Department of Gastroenterology and Hepatology, School of Medicine in Katowice, Medical University of Silesia, Medyków 14, 40-752 Katowice, Poland

**Keywords:** Vaspin, Adipose tissue, Hepatocellular carcinoma, Oxidative stress, Apoptosis signaling pathway, Hep-3B cells

## Abstract

**Background:**

Among adipose-derived factors, adipocytokines play roles as hormones and signaling mediators for apoptotic pathway. Among of them, vaspin, regulates the metabolism of adipose tissue itself as an endocrine organ, and stimulates adipocytes to maturation, differentiation, etc. Damaged adipocytes, present in obesity and hepatocellular carcinoma (HCC) respond with over-production of inflammatory cytokines. Such pro-inflammatory stimulation remains under adipokine control. Pro-inflammatory pathways are connected to oxidative stress and apoptosis, reported as co-existing with an elevated level of some adipokines in cancer cell lines. However, some hormones, such as vaspin, reduce apoptosis, have anti-inflammatory and anti-oxidative roles in cancer cell lines.

**Methods:**

Hep-3B cells were cytometrically evaluated under vaspin treatment for reactive oxygen species (ROS) and apoptosiss induction. The statistical significant changes to the untreated controls was calculated by T-tests (indicated at value *p* < 0.05).

**Results:**

Here we studied the production of reactive oxygen and nitrogen species in cells of HCC line Hep-3B after vaspin treatment. A decreased level of nitric oxide and superoxide anion 24 h after vaspin addition at 5 ng/ml was correlated with restricted, to the physiological level, apoptosis. A protective role of vaspin was displayed as enhanced cell viability and proliferation, which could be a poor prognostic in liver cancer.

**Conclusions:**

Apoptosis was suppressed after vaspin treatment, together with low levels of nitric oxide and superoxide anions.

## Background

Enhanced secretion of adipose-derived hormones termed adipokines or adipocytokines, like growth factors and pro-inflammatory cytokines, allows to focus on elements for studies of the pathogenesis of tumor growth, increased mobility and cell migration, and subsequently cancer metastasis [1, 2]. The adipokines could play a significant role in regulation of cell growth, proliferation, cell cycle, angiogenesis and also tumor growth and metastases [3]. One of the adipokines, leptin, is expressed in colorectal tumors with a greater expression in more aggressive tumors [4]. Cell motility is one of the most important factors that can affect both cell migration and invasion in cancer. There is probably a molecular and regulatory role for adipokines, also in cancerogenesis, migration and cancer progression. The possible mechanisms which clarify the associations between obesity and cancers are based on the promoting of growth signaling, inflammation, vascular disorders and microenvironmental dysfunctions [5–7].

Studies of the molecular mechanisms of actions of cytokines were done on a model cell line Hep-3B, originated from hepatoma [5]. This human HCC cell line has been reported as lacking a functional *p53* gene, so different physiological pathways, especially p53-dependent, could be defective or disturbed in that cell line [8]. Mutations of the *p53* gene are the most frequent in human cancers, also in hepatocellular carcinomas [9]. Lack of the *p53* gene also influences cellular death, e.g. apoptosis dependent on AKT/PTEN/FOXO4-pathways. Long-term hormonal treatments with visceral adipose tissue-derived vaspin presented a wide spectrum of activities for that molecule [10].

Aim of presented work, was to study one of the multiple modes of action of adipose tissue-derived hormones, an anti-apoptotic function of vaspin, and was examined in Hep-3B cells. Reactive oxygen species (ROS) were assessed with a particular emphasis on nitric oxide (NO), superoxide anion (•O_2_-), and overall ROS level estimated by 2′,7′-dichlorofluorescein diacetate (DCFH-DA) and a specific DNA-associated dye (CellROX Green). Oxidative stress, either induced by viral infections, inflammation, or external factors (*eg* ultraviolet or ionizing radiation), typically should result in cellular death through necrotic or apoptotic pathways. In p53 mutant cancer cell lines, this scheme is rather disrupted and cell death does not occur [9]. Cancer cell survival is promoted together with proliferation [9]. Some of the adipose tissue-derived hormones, like vaspin, protect p53 mutants against apoptosis activation [8], and the results presented in this study indicate a reduction of natural oxidative stress. Free radical scavenging in cells exposed to vaspin resulted in reduction of pro-oxidative apoptotic signaling pathways.

## Methods

### Cells

Human hepatocellular carcinoma (Hep-3B) cells from ATCC (Manassas, VA, USA) were a kind gift from Dr. Marek Rusin, from collections at the Maria Sklodowska-Curie Memorial Cancer Center and Institute of Oncology, Gliwice, Poland. Cells were grown in DMEM-F12 medium (PAA, Poland) with 10% (v/v) heat-inactivated fetal bovine serum (FBS) (EURx, Poland) and 10000 μg/ml streptomycin and 10000 units/ml penicillin) (Sigma-Aldrich, Germany), at 37 °C in a humidified atmosphere with 5% CO_2_. For flow cytometric measurements cells were seeded in 6-well plates (Falcon) at 10^5^ cells/well in 2 ml fresh medium and after 24 h the medium was replaced with fresh medium containing vaspin at 10, 5, 2.5, 1.25, 1 or 0.1 ng/ml. For MTS viability assays cells were seeded at 10^4^ cells/well in 96-well plates (Falcon) in 0.2 ml medium and after 24 the medium was replaced with fresh medium containing vaspin. Untreated controls were prepared for flow cytometry and MTS assays.

Vaspin was from Enzo Life Sciences (cat. No. ALX-201-360-C050) and dissolved in sterile PBS (PAA). Concentrated stock solutions (0.05 mg/ml) were stored at − 20 °C and working solutions were prepared in fresh growth medium.

### Apoptosis assays

Cells exposed to vaspin for 24 h were washed and collected by trypsinization. Cells were centrifuged (0.4 rcf, 3 min) and stained according to the Annexin-V apoptosis assay (Boncel et al., 2017). Cell pellets were dissolved in 50 μl cold Annexin-V labeling buffer and then 2.5 μl of FITC-labeled Annexin-V antibody was added (BioLegend) followed by 10 μl of propidium iodide (PI) solution (100 μg/ml; Sigma). After 20 min in darkness, 250 μl of Annexin-V labeling buffer was added and the samples were incubated on ice and in the dark for 15 min. Flow cytometric analysis (Aria III, Becton Dickinson) using the FITC configuration (488 nm excitation; emission: LP mirror 503, BP filter 530/30) and the PE configuration (547 nm excitation; emission: 585 nm) was performed immediately and at least 10,000 cells were counted. Cells were classified as necrotic (PI positive and Annexin-V negative; late apoptotic (PI positive and Annexin-V positive); early apoptotic (PI negative and Annexin-V positive); or normal (PI negative and Annexin-V negative) [11].

### MTS viability assays

Cells were incubated with vaspin for 24, 48 or 72 h, washed three times with PBS (PAA), and 20 μl of MTS solution (Promega) in 100 μl PBS (PAA) were added to each well according to the producer protocol [12]. The plates were incubated for 2–4 h until the color in the control wells had changed from light yellow to brown. The absorbance of formazan produced by live cells was measured at 490 nm using a microplate spectrophotometer (Epoch; BioTek) and is expressed as means ± SD from 3 experiments in triplicate and as fold changes of viability compared to untreated control cells.

### Cytometric measurements of reactive oxygen species and nitric oxide

Overall ROS levels were measured by flow cytometry using specific dyes, 2′,7′-dichlorofluorescin diacetate (DCFH-DA; Sigma) for reactive oxygen species (ROS), CellROX Green (Life Technologies) for superoxide anion (•O_2_-), or MitoSOX™ Red (Life Technologies) for mitochondrial superoxide and DAF-FM (Life Technologies) for nitric oxide (NO), as described previously [13, 14]. DCFH-DA, a cell-permeable non-fluorescent probe, converts into the highly fluorescent 2′,7′-dichlorofluorescein (DCF) upon deacetylation by intracellular esterases and oxidation by ROS. CellROX Green is also a cell-permeable, non-fluorescent probe which becomes highly fluorescent in the presence of superoxide anions and then binds to double-stranded DNA, mainly in the nucleus. MitoSOX is oxidized by mitochondrial superoxide but not by other ROS or reactive nitric species (RNS) to produce red fluorescence. DAF-FM diacetate is cell-permeable and is deacetylated inside cells to DAF-FM, which is converted to a fluorescent benzotriazole when it reacts with NO.

For flow cytometric measurement of ROS and NO, 300 μl of duplicate samples of cells in PBS were stained either with DCFH-DA (30 μM), CellROX Green (2.5 μM) for ROS detection, MitoSOX Red (2.5 μM) for superoxide anions, or DAF-FM (2.5 μM) for nitric oxide (NO). After incubation in darkness at 37 °C for 30 min the cells were washed with PBS and kept in the dark for 15 min on ice (DCFH-DA and CellROX Green) or at room temperature (MitoSOX Red and DAF-FM). Fluorescence was measured using the FITC configuration for DCFH-DA, CellROX Green and DAF-FM or the PE configuration for MitoSOX Red [11]. At least 10,000 cells were counted. The results were analyzed using the free software FlowingSoftware 2.5.0 (Perttu Terho, Turku Centre for Biotechnology, University of Turku, Finland) and are presented as mean fluorescence.

### Statistical analyses

Results are presented as means ±SD from three separate experiments, performed in six replicates for cytotoxicity and triplicates for cytometric assays. The experimental means were compared to those for untreated cells collected in parallel. The results were analyzed using MS Office ver. 2.5.0 and MS Excel 2007. Statistical significance vs the control was calculated by T-tests and *p* < 0.05 is indicated by*.

## Results

After growth of Hep-3B cells in the presence of vaspin the fraction of apoptotic cells was reduced (Fig. 1a, b and c). Within the apoptotic fraction, apoptosis assays together with DNA staining distinguished necrotic from apoptotic cells and early from late apoptosis [11]. In control cultures the apoptotic fraction did not exceed 10% of the total cells for early and 15% for late apoptosis, and necrosis was almost undetectable (Fig. 1c). Vaspin at 10 ng/ml reduced the frequency of total apoptotic cells significantly after 24 h, showing that a mechanism protecting cells against apoptosis was activated.

**Fig. 1:** Example of flow cytometry apoptosis dot plots (**a**), where Iodium Propide positive stained mined necrotic cells (PI + and FITC -); Iodium Propide positive and Annexin-V positive mined apoptotic cells (PI + and FITC +). Apoptotic (**b**) and apoptotic and necrotic cells (**c**) after growth for 24 h with vaspin. * values statistically significant vs control; T-test (*p* < 0.05)

This conclusion was supported by assays of cell proliferation and survival. Compared to untreated control cells, the best viability was observed at 48 h (Fig. 2a). After 24 h with vaspin a slightly increase of viability was observed at doses of 5–10 ng/ml, and at 1 ng/ml the viability increased almost 1.5-fold in comparison to the control (Fig. 2b).

**Fig. 2:** Viable cells measured by MTS assays during growth with vaspin(**a**); fold-change of the number of viable cells relative to controls (**b**). *values statistically significant vs control; t-test (*p* < 0.05)

The activation of apoptosis is often correlated with cellular oxidative stress, either internally or externally induced. Normal functions of cells cause physiological production of free radicals, for example superoxide anions by mitochondrial complexes I and III of the cytochrome chain [15]. Free radicals are also present as signaling molecules produced by enzymes such as the seven membrane-bound NADPH-dependent oxidases (Nox1–5 and Duox1–2) [16, 17]. Among short-lived molecules, nitric oxide (NO) is an important signaling molecule [14].

Cytometric measurements showed fluctuations of NO level after 24 h exposure to vaspin. At 2.5 ng/ml of vaspin NO increased significantly compared to the untreated control (Fig. 3a and b), while at 5 ng/ml its level decreased. A second, significant increase in the level was induced by vaspin at 10 ng/ml for 24 h (Fig. 3b). These fluctuations seemed to be crucial for apoptotic pathway inhibition (Fig. 1) and enhanced viability and proliferation (Fig. 2). The level of superoxide anion, measured using the specific probe MitoSOX, decreased after 24 h of incubation with 2.5–5 ng/ml vaspin (Fig. 3c and d). The physiological level of superoxide anion was rather stable at other vaspin concentrations, and comparable to the control. At the highest dose of vaspin (10 ng/ml) the level of •O_2_- returned to a value slightly higher than the control (Fig. 3d).

**Fig. 3:** Flow cytometry histograms and levels of NO (**a** and **b**) and superoxide anion (**c** and **d**) after 24 h growth with vaspin, measured by DAF-FM and MitoSOX Red staining, respectively. *values statistically significant vs control at *p* < 0.05. Positive control from cells treated for 5 min with H_2_O_2_ at concentration of 100 μM

Flow cytometry measurements of NO and •O_2_- indicated on a strong relationship between the low levels observed at 5 ng/ml vaspin and inhibition of apoptosis (Figs. 1, 2). These low levels were significant in comparison to those in untreated controls during 24 h of incubation in the same conditions (Fig. 3). So, inhibition of apoptosis at 5 ng/ml of vaspin is related to decreased levels of signaling molecules such as NO and •O_2_- (Fig. 3). Recovery of NO and •O_2_- to physiological levels, and even an elevation over the control level at higher doses of vaspin, did not change its protective activity. There appears to be a switch which is turned on at lower doses of vaspin (2.5 ng/ml) but activated by higher than control levels of NO, and at lower doses of vaspin (1 ng/ml) is activated by higher than control levels of •O_2_- (Fig. 3). Once initiated, an anti-apoptotic cascade is maintained at higher vaspin concentrations (5–10 ng/ml) (Figs. 1 and 3). The lowest levels of NO and •O_2_- at 5 ng/ml of vaspin inhibited apoptosis efficiently (Figs. 1 and 3).

To better understand the role of ROS in induction/inhibition of the apoptosis pathway, further measurements of ROS were performed. Specific staining of ROS using the probes DCFH-DA and CellROX Green did not detect significant changes in free radicals level. At the lowest vaspin dose (0.1 ng/ml) the ROS level after 24 h of incubation decreased only slightly in comparison to untreated controls (Fig. 4). At 1–10 ng/ml of vaspin the level of ROS recovered to the control level as assayed by either probe (Fig. 4). Flow cytometry measurements discriminated between overall and DNA-associated ROS, but did not explain the role of global ROS in cells after hormonal exposure. The level of ROS was stable during 24 h of incubation, without any spectacular changes related to the vaspin dose (Fig. 4). Inhibition of the apoptosis pathway after vaspin treatment was connected to lowered NO and •O_2_- levels, rather than to the stable level of ROS overall (Figs. 1, 3 and 4).

**Fig. 4:** Levels of intracellular ROS after growth for 24 h with vaspin assayed by DCFH-DA (**a**) or by CellROX Green (**b**). Experimental values were not significantly different from controls; T-test (*p* < 0.05)

## Discussion

Processes such as improved viability, proliferation, and survival after inhibition of apoptosis in cancer cells depend on external and internal cross-talk between signaling pathways and many factors and hormones, including vaspin [10, 18–20]. The present studies were done to better understand the multiple roles of vaspin, an adipokine derived from adipose tissue. Vaspin protected human hepatocellular carcinoma cells against oxidative stress and apoptosis. Reactive oxygen species, nitric oxide, and superoxide anion appear to be involved in this anti-apoptotic activity.

### Adipose tissue delivers regulatory factors

In the human body, adipose tissue plays the role of a systemic endocrine organ through whole-body energy regulation and glucose homeostasis [21]. They produce numerous bioactive factors such as adipokines which play roles of cytokines in metabolic disorders including obesity and related diseases, and since two decades visfatin, leptin, hepcidin, adiponectin, vaspin, apelin, chemerin, omentin, and others have been discovered and extensive studied [21–24]. Adipose tissue is known as brown (BAT) and white (WAT), associated respectively with thermoregulation and obesity in animals and adipocyte maturation and regulatory factor delivery [25]. Connections within adipose tissue depend on the regulatory factors which they produce (hormones, cytokines) or on processes occurring in the body (viral infections, inflammation) (Fig. 5). External factors delivered with nutrition via the digestive tract also interact with adipose tissue, directly or through induced processes (e.g. liver injury and inflammation after alcohol intake or heavy metal pollution) [3, 26–28]. An interaction with adipose tissue-delivered factors seems to be crucial and very important for pathogenic processes such as human hepatocellular carcinoma development and progression (Fig. 5).

**Fig. 5:** Interactions between natural and artificial agents (viruses, hormones, biomolecules, and nanoparticles) in liver cancer development

### Vaspin enhances hepatoma cell viability and proliferation

The protective activity of vaspin on Hep-3B cells was confirmed by Annexin-V apoptosis assays, where apoptosis was suppressed in a dose-depended manner (Fig. 1). The fraction of normal cells (PI negative and Annexin-V negative) in the population increased to almost 100% at 5–10 ng/ml vaspin (Fig. 1), and viability measured by MTS assays increased (Fig. 2). Some adipokines are known as protectors of cancer cells because they play a role of promoters in cancer cell progression and enhance metastasis through stimulation of cell proliferation and migration [4]. Adipose-derived hormones, cytokines stimulating inflammatory process, and growth factors are responsible for the pathogenesis of tumor growth [4]. Only a few studies suggest a stimulatory effect of vaspin on proliferation of cancer cells [4, 29, 30]. An elevated vaspin level was reported in colorectal cancer [31] but a lower level in endometrial cancer [32]. Vaspin also increased the proliferation of rat insulinoma cells [33]. Angiogenesis, new blood vessels formation, seems to be essential in cancer development and progression. Vaspin was positively related to intensity of angiogenesis in chronic hepatitis [24] via association of adipokines with angiogenesis. The main risk factor of HCC in chronic liver diseases is advanced fibrosis/cirrhosis, which is strictly associated with angiogenesis intensity [7, 34]. Vaspin serum levels and mRNA liver expression were found to be increased in patients with advanced fibrosis or cirrhosis in the course of chronic hepatitis [35, 36]. Pointing to these results, vaspin plays pivotal role in HCC development. Increased vaspin levels and expression in advanced liver disease may protect cancer cells against apoptosis and facilitate their proliferation.

### Role of adipokines in regulating oxidative stress

Physiological oxidative stress results from endogenous processes like mitochondrial oxidative phosphorylation and the electron transport chain, lipid β-oxidation, peroxisome activity, and protein degradation, and signal transduction via free radicals which produce reactive oxygen and nitrogen species in living cells [37, 38]. Imbalance in production and scavenging of free radical leads to numerous metabolic disorders including cancer stem cell activation and cancer development (reviewed in [39]). Adipose tissue produces factors such as visfatin which impact on free radical levels through influencing the enzymatic systems responsible for ROS production or inactivation [4, 40–42]. In HCT116 colorectal cancer cells oxidative stress was decreased by another adipokine, visfatin, and ROS levels decreased, but apoptosis increased and viability was reduced, so there visfatin showed pro-apoptotic activity uncorrelated with the ROS level [41]. On the other hand, in Me45 melanoma cells visfatin increased oxidative stress and ROS due to its pro-inflammatory action in increasing production of interleukins IL-6 and IL-8 [42]. Studies on Huh-7 liver HCC cells showed association between cell migration and elevated ROS level via TNF-α-activated NF-ĸB signaling [43]. The pro-oxidative activity of vaspin was tested in human endothelial EA.hy926 cells, and unlike visfatin it protected them from inflammation by inhibiting NF-ĸB signaling [20]. In rodents, vaspin inhibited TNF-α-induced ROS generation in rat vascular smooth muscle cells and showed anti-oxidant protection [19].

Although in Hep-3B cells no significant elevation of global ROS level during 24 h of vaspin treatment was observed in our study (Fig. 4) the role of particular free radicals and signaling molecules, NO and •O_2_-, appeared to be important in modulating apoptotic pathways. After 24 h of vaspin treatment the NO level fluctuated significantly in a dose-dependent manner (Fig. 3), but oxidative stress was rather weak this might be crucial for limiting apoptosis. Superoxide anion levels also fluctuated, with a minimum at 5 ng/ml of vaspin. The decreased level of both NO and •O_2_- at 5 ng/ml of vaspin resulted rather from suppression of physiological oxidative processes (Fig. 3). Resveratrol was reported to be an antioxidant in rat adipose tissue in type 2 diabetes because of vaspin gene down-regulation, that mined vaspin absence resulted with oxidative stress reduction [44]. The explanation for vaspin’s impact on mitochondrial activity remains unclear, however, reduced production of superoxide anions was observed in our study (Fig. 3). The role of NO in vaspin-treated hepatoma cells should be rather explained as a pro-inflammatory signaling molecule. Modulation of its level appeared to result from activation of inflammation processes and their reduction after vaspin treatment (Fig. 3). Consequence for that could be also elevated pro-inflammatory cytokines production and vaspin inhibited that inflammatory process [18, 20, 45]. NO was correlated to the serum vaspin level in type 2 diabetes patients with nephropathy, where vaspin had a stimulatory effect through the activation of NO synthase [46]. We conclude that in Hep-3B cells an elevated level of vaspin results in modulation of the level of NO and •O_2_-, with a significant depression at 5 ng/ml of vaspin (Fig. 3). In consequence, mitochondrial activity is reduced because the level of superoxide anion decreases below the control value. Generally, in Hep-3B cells vaspin reduced the physiological level of oxidative stress (Fig. 4) but did not influenced it greatly. Reduction of ROS, with specific reduction of NO and •O_2_-, could restrict pro-inflamatory processes in cancer cells leading to better viability and proliferation (Figs. 1, 2) [47].

### Vaspin down-regulates apoptotic pathways in Hep-3B cells

Our observations on the effects of vaspin on Hep-3B cells can be summarized as a restriction of apoptosis resulting from limitation of mitochondrial free radicals, especially superoxide anions (Fig. 3). A decreased level of NO results in an anti-inflammatory effect after vaspin treatment at 5 ng/ml (Fig. 3). Perhaps, pro-apoptotic signals in the canonical mitochondrial apoptosis pathway are suppressed by vaspin, and lower levels of ROS and NO are correlated with inhibition of cell death (Figs. 1 and 4). All ROS-dependent pathways should be under particular consideration, especially in HCC, including the p53-null Hep-3B cell line. In p53 mutants also receptors for apoptosis mediators, such as NF-κB, Bcl-2 or Bcl-XL could be disrupted and apoptosis propagation stopped [48]. Vaspin could be a good mediator for anti-apoptotic and anti-oxidative status influenced by lowered level of nitric oxide and superoxide anion. A different role for vaspin was suggested in patients with nonalcoholic fatty liver disease, where a chronic inflammatory state was observed. Although the vaspin serum level was low the pro-inflammatory cytokines level was elevated [49, 50]. Moreover, vaspin levels increased in definite nonalcoholic steatohepatitis when compared to simple steatosis and in patients with hepatocyte ballooning, which may reflect oxidative stress and mitochondrial disfunction in hepatocytes [7]. The role of vaspin, either anti/pro-inflammatory, anti/pro-oxidative, or anti/pro-apoptotic is still unclear, but in Hep-3B cells it is rather protective (Fig. 6). Elevated serum concentrations of vaspin are associated with obesity and impaired insulin sensitivity in humans and it has therefore been postulated that increased vaspin expression and secretion could represent a compensatory mechanism associated with obesity, severe insulin resistance, and type 2 diabetes [51].

**Fig. 6:** Compensatory mechanisms associated with obesity and the anti-apoptotic and protective actions of vaspin in Hep-3B cells

## Conclusions

Apoptosis was suppressed after vaspin treatment, together with low levels of nitric oxide and superoxide anions.

## Data Availability

The datasets used and analyzed during the current study are available from the corresponding author on reasonable request.

## Abbreviations

AKT: Serine/Threonine Kinase
BAT: Brown adipose tissue
DCFH-DA: 2′,7′-dichlorofluorescein diacetate
Duox: dual NADPH-dependent oxidases
FBS: Fetal bovine serum
FOXO4: Forkhead box protein O4
HCC: Hepatocellular carcinoma
Hep-3B: Human hepatocellular carcinoma
NF-ĸB: Nuclear factor kappa-light-chain-enhancer of activated B cells
NO: Nitric oxide
Nox: NADPH-dependent oxidases
PI: Propidium iodide
PTEN: Phosphatase and tensin homolog
ROS: Reactive oxygen species
TNF-α: Tumor necrosis factor alfa
WAT: White adipose tissue
